The article "Effects of Hypoxia-Inducible Factor 1 (HIF-1) Signaling Pathway on Acute Ischemic Stroke" was retracted in 2023. Reasons: signs of a paper mill; compromised peer review; unreliable results or conclusions.

# Effects of Hypoxia-Inducible Factor 1 (HIF-1) Signaling Pathway on Acute Ischemic Stroke

**DOI:** 10.1155/2022/1860925

**Published:** 2022-10-14

**Authors:** Guoliang Li, Liang Tao, Hui Wu

**Affiliations:** ^1^Department of Neurosurgery, People's Hospital of Dongxihu District, Wuhan, Hubei 430040, China; ^2^Department of Neurosurgery, Wuhan Third Hospital, Tongren Hospital of Wuhan University, China; ^3^Department of Traditional Chinese Medicine, Wuhan NO.1 Hospital, 215 Zhongshan Avenue, Qiaokou District, Wuhan, China

## Abstract

**Background:**

Epidemiological surveys show that a large number of cerebrovascular diseases occur in China every year, and among these cerebrovascular diseases, ischemic diseases are predominant. Ischemia leads to irreversible degenerative necrosis of a large number of brain neurons and severe neurological deficits.

**Aims:**

This study is aimed at exploring the mechanism of the major regulatory effect of hypoxia-inducible factor 1 (HIF-1) pathway on proangiogenesis and providing new ideas for the treatment of ischemic stroke.

**Materials and Methods:**

The rats were randomly divided into normal and ischemic control groups, and the ischemic control group was subjected to the middle cerebral artery occlusion (MCAO) cerebral ischemia model by the wire embolization method, and the rats were executed in batches at 6 h, 1 d, and 3 d after ischemia-reperfusion, and the brain tissue specimens were taken for examination to investigate the effect of hypoxia-inducible factor 1 (HIF-l) signaling pathway on acute ischemic stroke.

**Results:**

At 3 d, the number of VEGFR2 positive cells increased significantly, and there was a significant difference compared with the control group (*P* < 0.05). At 3 d, the number of HIF-1*α*-positive cells increased significantly, and there was a significant difference compared with the control group (*P* < 0.05). The number of Hes1+factor VIII positive cells in the ischemic cortex increased significantly on the 1st and 3rd day, and there was a significant difference compared with the control group (*P* < 0.05). The expression of Hes1 protein was significantly lower than the normal level after 6 h of ischemia, and the protein expression was significantly increased at 1 d and 3 d after ischemia (*P* < 0.05).

**Conclusion:**

By detecting the expression changes of Hesl+factor VII in the ischemic area, the results show that ischemia and hypoxia activate the HIF-1, making the HIF-l the main regulatory pathway in the process of angiogenesis after ischemia.

## 1. Introduction

With the in-depth study of the pathophysiology of cerebral ischemic area, it is recognized that there is a penumbra after ischemia, that is, the relative ischemic area around the ischemic core area [1]. In the penumbra area, due to incomplete ischemia due to the supply of collateral circulation, a large number of neurons only undergo reversible degeneration. This reversible degeneration provides an opportunity to rescue as many neurons as possible in future treatments [2]. If the formation of new blood vessels in the ischemic area can be promoted to restore local blood flow as soon as possible, it is not only beneficial to rescue reversibly degenerated neurons but also provides a good microenvironment for the survival, proliferation, and functional remodeling of neural stem cells in the subsequent functional repair. Treatment of stroke can minimize neurological deficits and improve prognosis [3]. Clinical research data show that the prognosis of patients with high-density of new capillaries in the area of cerebral ischemia injury is significantly better than that of patients with low-density, so it can effectively promote the formation of local blood vessels in the ischemic area as soon as possible to restore the blood reperfusion of ischemic brain tissue. The treatment of blood stroke is of great significance [4].

Neovascularization refers to the process of sprouting and forming new functional blood vessels on the basis of the original vascular network, which can be seen in many pathological and physiological processes [5]. In the process of neovascularization, the expression and synergistic effect of numerous vascular growth factors are required, the most important of which is vascular endothelial growth factor (VEGF) [6]. VEGF is one of the target genes directly regulated by HIF-1, and the two are closely related to the process of angiogenesis after ischemia. In ischemic brain tissue, both are expressed on neurons with the same expression phase [7]. HIF-1 is a transcription factor discovered during erythropoietin gene expression studies in hepatocytes and transgenic animals [8, 9]. So far, more than 100 target genes have been found to directly act on HIF-1, which are involved in the processes of angiogenesis, apoptosis, cell proliferation, and energy metabolism. Hypoxia activates HIF-1 in ischemic stroke and induces HIF-1 related processes. Target genes are transcribed and produce corresponding biological effects [10]. Animal models of ischemia have confirmed that HIF-1 protein can promote the formation of new blood vessels. Even after the removal of the oxygen-dependent degradation region, HIF-1 protein can still activate its downstream target genes to generate a large number of vascular tissues [11]. After hypoxia, HIF-1 not only affects the expression of angiopoietin, platelet growth factor, etc., but also directly acts on downstream target genes such as VEGF to participate in angiogenesis, making it a core regulator of angiogenesis after hypoxia [12]. Further study of its mechanism is that HIF-1 binds to the VEGF site under hypoxic conditions to enhance the expression of VEGF promoter, significantly increase the transcriptional activity of VEGF, and promote angiogenesis [13]. It can be seen that HIF-1 plays an indispensable role in the regulation of VEGF during angiogenesis under hypoxia.

## 2. Material and Methods

### 2.1. Research Object

Twenty clean-grade adult (9 weeks) male Sprague-Dawley (SD) rats weighing 250-280 g were selected, and the experimental rats were randomly divided into sham-operated, 6 h, 1 d, and 3 d postischemic groups, with 5 SD rats in each group. The rats with cerebral ischemia were executed at the corresponding time points of 6 h, 1 d, and 3 d after cerebral ischemia-reperfusion, respectively. The rats in the sham-operated group only did the same surgical operation without treating the carotid artery, and the rest treatments were the same for both.

*Sterilization:* The glass instruments used were soaked in sulfuric acid and potassium dichromate cleaning solution for 24h, then washed thoroughly, then rinsed with triple distilled water, dried in the oven at 60°C, and then sterilized by dry heat at 160°C for 2 h; the plastic equipment used were cleaned, rinsed with triple distilled water, dried at 60°C, and then autoclaved at 120°C; all metal surgical instruments were sterilized by immersion in glutaraldehyde.

*De-RNAse Treatment:* EP tubes, gun tips, and other disposable supplies were treated with 0.1% DEPC water overnight, dried, and then autoclaved at 120°C; reagents were prepared in newly opened bottles or DEPC water; metal, glass, and other supplies were sterilized by dry baking at 250 C for 4 h.

### 2.2. Experimental Animal Inclusion Criteria

The following signs were observed after awakening from anesthesia in the MCAO model, and those who showed the following signs indicated the success of the model: Horner's sign on the right side and neurological deficit on the left limb and neurological function score according to the Zea Longa 5-point scale: 0: normal, no symptoms of neurological damage; 1: unable to fully extend the contralateral front paw; 2: turn to the left when walking; 3: lean to the opposite side when walking; 4: unable to walk spontaneously, loss of consciousness. Animal models were included if they scored 1 – 3.

### 2.3. Methods

*Ischemic Injury Model*. The focal ischemic injury model of middle cerebral artery embolism was made by referring to the modified Longa and Nagasawa method. The brief steps are as follows: weigh 250-280 g of SD rats, rats were sacrificed intramuscularly at 2 mg/kg xylazine plus 10 mg/kg ketamine, and inject pentobarbital at the same time. Limbs and head were fixed supine on the operating table. Cut off the neck hair, sterilize the skin, make a longitudinal incision in the middle of the neck, and cut the skin to expose the right common carotid artery, internal carotid artery, and external carotid artery. Under the operating microscope, the anterior superficial and deep fascia of the neck was incised to expose the anterior trachea muscle group, which was separated to the depth between the angle formed by the anterior tracheal muscle group and the right sternocleidomastoid muscle. Next step is free the common carotid artery, internal carotid artery, and external carotid artery (be careful not to damage adjacent important nerves and branches) and ligate the proximal common carotid artery and the distal external carotid artery with silk thread, and the internal carotid artery is temporarily blocked by arterial clips. A V-shaped incision was made in the proximal wall of the external carotid artery, and a self-made 4-0 thread plug (about 3 cm in length, with a smooth sphere with a diameter of 0.3 mm at the tip) was inserted into the ordinary carotid artery through the incision first. The next step is insert a 4-0 wire plug (about 0.3 mm in diameter) into the common carotid artery through the incision, then completely incise the external carotid artery, tie the reserved wire on the external carotid artery A, and make sure that the wire plug is not too large when inserted resistance. After that, loosen the arterial clamp, slightly return the bolt at the bifurcation of the common carotid artery, and slide it into the internal carotid artery A. The next steps is slowly enter the middle cerebral artery without resistance, then block the blood supply of the middle cerebral artery, and then stop the insertion when the elastic resistance is felt, and the insertion length is about 18 ± 0.5 m from the bifurcation of the common carotid artery; after that, fix the bolt and apply a simple bandage incision. After blocking the blood supply of the middle cerebral artery for 2 hours, the neurological function of the awake rats was scored, and the rats were anesthetized again. And the rats were anesthetized again for internal carotid artery reperfusion. The cervical incision was sutured and returned to the cage. Rats in the sham operation group only had free blood vessels, and other treatments were the same as those in the operation group. The rectal temperature of SD rats was maintained between 36.5-37.0°C throughout the surgery. SD rats in each group were sacrificed, and the ischemic cortical brain tissue was preserved. The procedure was as follows: rats were sacrificed intramuscularly at 2 mg/kg xylazine plus 10 mg/kg ketamine, and the heart was perfused with 500 ml of sterile saline to isolate intact brain tissue. After that, place the brain tissue at 20°C for 30 min. Approximately 100 mg of each brain tissue was excised with a deribonuclease-treated razor blade from the affected cortical area before and after the bregma and divided into two deribonuclease-treated 1.5 ml EP tubes and stored in a refrigerator at 80°C.

5 frozen sections of each brain tissue were randomly selected from each experimental group at each time point, and the expression of VEGFR2 in the ischemic cortical area was detected by immunohistochemical staining, and the specific steps were the same as those for HIF-1*α* immunofluorescence staining and briefly described as follows: rabbit anti-rat VEGFR2 antibody (1 : 100) was added to the brain tissue sections in 60 ul drops, completely covering the brain tissue, at 4°C. The sections were wet boxed overnight, and FITC-labeled goat anti-rabbit IgG (1 : 200) 60 ul was added dropwise on the next day, and the reaction was performed at 37°C for 50 min, protected from light. Glycerol-sealed slices were observed under fluorescence microscope and photographed.

#### 2.3.1. *Result Determination:* the cytoplasm cytosol of VEGFR2-positive cells showed green fluorescence under fluorescence microscope. *Counting:* 5 nonoverlapping fields of view were randomly selected in the ischemic cortical area of each section at ×400 cell counting, and the average number of positive cells in each field of view was taken for each brain tissue.

#### 2.3.2. Detection of HIF-1

5 frozen sections of each brain tissue were randomly selected from each experimental group at each time point, and the expression of Hs1 and microvessel density in vascular endothelial cells in ischemic cortex was detected by double immunohistofluorescence staining with HIF-1+factor VIII. The specific steps are the same as HIF-1*α* factor immunofluorescence staining: mix mouse anti-rat Hes1 antibody and rabbit anti-rat factor VVII antibody in 0.01 M PBS, so that the final concentration of both antibodies is 1 : 100, take 60ul of the mixture and add on brain tissue sections, react at 4°C for 24 hours; mix TRITC-labeled bovine anti-rabbit IgG and FITC-labeled goat anti-mouse IgG in 0.01MPBS, so that the final concentration of the two antibodies is 1 : 200, take and mix Add 60 ul of the solution to the brain tissue section and react at 37°C for 50 minutes in the dark, and add 50 ul of 1% DAPI solution dropwise and react in the dark for 5 min at room temperature. After mounting with 50% glycerol, observe and take pictures under a fluorescence microscope. The results showed that the cytoplasm of vascular endothelial cells showed red fluorescence under the fluorescence microscope, the cytoplasm of Hs1-positive cells showed green fluorescence, and the nuclei of all cells showed blue fluorescence after DAPI staining. *Counting:* 5 nonoverlapping visual fields were randomly selected in the ischemic cortex of each slice to count Hes1-positive vascular endothelial cells, and the average number of Hs1-positive endothelial cells in each visual field of each brain tissue was taken.

### 2.4. Statistical Analysis

All statistical data in this study were entered into Excel software by the first author and the corresponding author, respectively, and the statistical processing software was SPSS25.0 for calculation. The mean ± standard deviation ($\bar{x}$±*s*) was used to represent the measured value of the measurement data and compared with the analysis of variance between groups. Count data were expressed as a percentage (%) and compared with *χ*^2^ analysis. Repeated measures analysis of variance between groups was used to measure the measurement expressed as mean ± standard deviation ($\bar{x}\pm \text{s}$). Count data expressed as a percentage (%) were tested by *χ*^2^. Included data that did not conform to a normal distribution were described by M (QR), using the Mann–Whitney test. All statistical tests were two-sided probability tests, and the statistical significance was *P* < 0.05.

## 3. Results

### 3.1. Expression of HIF-1

There was only a small increase in the number of HIF-1*α* positive cells in the cortical area after 6 h and 1 d of cerebral ischemia-reperfusion, and the difference in the number of HIF-1 positive cells after 6 h and 1 d was not statistically significant compared with the control group (*P* > 0.05); however, by 3 d, there was a significant increase in the number of HIF-1*α* positive cells, which was statistically significant compared with the control group (*P* < 0.05). See Figure 1.

### 3.2. Expression of VEGFR2

The number of VEGFR2-positive cells in cortical areas increased in a few after 6 h and 1 d of cerebral ischemia-reperfusion, and the difference between the number of VEGFR2-positive cells after 6 h and 1 d compared with the control group was not statistically significant (*P* > 0.05); however, by 3 d, the number of VEGFR2-positive cells increased significantly, and there was a statistically significant difference compared with the control group (*P* < 0.05). See Figure 2.

### 3.3. Changes in Microvessel Density

After 6 hours of cerebral ischemia-reperfusion, the number of Hes1+factor VIII positive cells in the ischemic cortex was lower than normal, and there was a statistical difference between the control group and the 6 h group by *t*-test (*P* < 0.05). After 1 d and 3 d ischemic cortex the number of Hes1+factor VIII positive cells in the area increased significantly, compared with the control group, there was a significant difference (*P* < 0.05). See Figure 3.

### 3.4. Test Results

The expression of HIF-1*α* protein in ischemic cortex was changed at 6 h, 1 d, and 3 d. The expression of HIF-1 was almost the same as normal after 6 h of ischemia. The expression of HIF-1*α* protein increased significantly after 1 d and 3 d of ischemia, but the expression of HIF-1*α* was significantly increased after 1 d and 3 d of ischemia. The expression of notch1 protein gradually increased in the cerebral cortex at 6 h, 1 d, and 3 d after ischemia and reached a peak at 3 d, while the expression of Hes1 protein first decreased and then increased. After 6 h of ischemia, the Hes1 protein expression was significantly lower than the normal level, and then the protein expression increased significantly at 1 d and 3 d. See Figure 4.

## 4. Discussion

There is still little progress in the treatment of ischemic stroke, which is still based on symptomatic, neurotrophic, thrombolytic, and anticoagulant treatments with poor prognosis and many residual complications [14]. With the deepening of the understanding of the pathophysiology of the ischemic zone of brain tissue, the concept of cerebral ischemic semidark zone was proposed, and people turned to advocate early restoration of blood flow to save the dying cells in the semidark zone and improve the prognosis of treatment [15]. Newly generated microvessels not only provide blood supply to the ischemic zone but also induce the release of various trophic factors, which are beneficial for neurological recovery. It has been observed in clinical practice that the higher the number of microvessels in the brain tissue of ischemic stroke patients, the longer their poststroke survival time [16]. VEGF is an early and well established vascular growth factor that has been widely used in ischemic diseases, and previous studies have demonstrated that the administration of exogenous vascular growth factor stimulates neurological recovery in ischemic areas. The study of other VEGF-related factors and signaling pathways has further improved the understanding of the process of angiogenesis and provided new ideas for the treatment of ischemic stroke [19].

Both subunits have a base helix loop helix and PAS structure and belong to the bHLH-PAS family [20]. The subunits are located in the cytoplasm, and their concentration levels are correlated with low oxygen concentration levels, while the B subunit is a constructive expression, independent of oxygen concentration, mainly related to maintaining HIF structural stability and dimerization activity conformational shift [21]. Hypoxia-induced production of HIF-1 on neovascularization is currently recognized by the following mechanisms of action: preparation for angiogenesis by synthesizing vasodilation and upregulation of VEGFE and ligand expression to increase vascular permeability [22]. Upregulation of metalloprotein hydrolase activity and degradation of the extracellular matrix provide an environment for cell survival [23]. HIF-1 acts on VEGF to induce migration and proliferation of vascular endothelial cells, binds angiopoietin, and promotes vascular sprout formation [24]. Through the action of VEGF, angiopoietin and integrin, single vessel bud lumen anastomoses with each other forms a vascular network and finally acts on stromal cells through platelet-derived growth factor and angiopoietin 1 to wrap around the neovascularization to form mature vessels [25]. Through the above mechanism of action, it makes HIF-1 a central regulator of posthypoxia vascular neogenesis. *α* is the active regulatory unit of HIF-1, which includes two important structural domains: the oxygen-dependent degradation structural domain, which regulates the stabilizing effect of HIF under oxygen concentration [26] and the two transcriptional activation structural domains, one each at the N- and C-termini. C-TAD regulates gene transcriptional activity, while N-TAD is the domain of action that forms heterodimers with HIF-1*α* and binds DNA cis-response elements [27]. Three sequence homology a-subunits have been identified: HIF-1*α*, HIF-2*α*, and HIF-3*α*. Hypoxia is the predominant HIF-1 expression apoptotic factor, and hypoxia-activated HIF-1*α* binds to HIF-1*β*, translocates into the nucleus, cross-links to hypoxic response elements in the regulatory region of target genes, and induces gene expression [28]. Under normoxic conditions HIF-l*α* is hydroxylated by prolyl hydroxylase and acetylated by acetyltransferase, and the hydroxylated and acetylated HIF-1*α* is then bound to the Von Hippel-Lindau (pVHL) protein and degraded by ubiquitination [29]. Also because the asparagine hydroxylation of HIF-1*α* affects its binding to the hypoxic response element of the target gene enhancer thereby inhibiting the transcription of downstream target genes, and more than 100 target genes have been found to be directly acted upon by hypoxia-inducible factors, which are involved in processes such as angiogenesis, cell regulation, cell proliferation, and energy metabolism [30]. Due to the importance of VEGF for neovascularization, the relationship between HIF and VEGF after hypoxia has been extensively studied in-depth [31]. In a neonatal mouse model of MCA 1.5 h, it was found that the positive expression of HIF-1 increased after 4 h of ischemia, peaked at 6 h, and started to decrease after 24 h, mainly expressed on neurons, while it was observed that VEGF mRNA appeared to be expressed in brain tissue after 2-4 h, declined after 6 h, and returned to normal levels at 24 h, while the site and temporal phase of VEGF protein expression were the same as those of HIF-1*α* [32]. In a model of cerebral ischemia caused by cardiac arrest, a significant increase in HIF-1 was detected after 1 h of reperfusion, and VEGF mRNA and VEGF protein increased at 12-46 h and 24-46 h and persisted until 7 d later, respectively [33]. Rapid expression of HIF-1 was also observed early in mice reischemic after hypoxic preconditioning, while its downstream gene products EPO and VEGF were also abundantly expressed after 6 h [34]. Some studies for the expression of HIF-1 after cerebral ischemia have suggested in the literature that the increase in its expression is induced by postischemic hypoxia [35]. The peak of HIF-1*α* expression after ischemia was observed at 3 d, while some scholars observed the peak of HIF-l*α* expression after low pressure cerebral ischemia at 48-96 h. Our experiment also observed an increase in HIF-1 expression after cerebral ischemia, and the results were basically similar to the literature [36]. The expression of HIF-1*α* increased after 6 h of ischemia-reperfusion, and the number of positive cells reached a peak at 3 d after ischemia. We observed that HIF-1*α* protein expression increased significantly on day 1 and day 3, but the peak appeared on day 1. The expression of VEGFR2 positive cells was also observed in a gradual increase, with the strongest expression at 3 d. For the peak of HIF-1 expression after ischemia, there are various scenarios appearing among different literature, for the delayed peak of HIF-1*α* expression after simple cerebral ischemia; this phenomenon has not been clearly explained in the literature, which may be related to a combination of factors such as induction of HIF-1 by rehypoxia after ischemic tolerance and induction of HIF-1*α* expression by inflammatory factors in response to tissue inflammation after ischemia [37]. Postischemic hypoxia HIF-1 exerts a regulatory effect on VEGF and affects angiogenesis [38]. With the in-depth study, it has been recognized that the apoptotic mechanism of HIF-1 on VEGF expression is as follows: activation of HIF-1 into the nucleus directly binds to HRE to activate VEGF genes and induce transcription [39]. HIF-1 upregulates the transcription of VEGFR1, and HIF-1 acts on specific sites of VEGF mRNA and increases its stability to ensure VEGF expression [40].

We learned from the results of this study by detecting the changes in the expression of Hesl+factor VII in the ischemic area, the results show that ischemia and hypoxia activate the HIF-1 signaling pathway, and with the increase of HIF-1 expression, it can effectively promote the formation of new blood vessels. The same point between the study and previous studies is that cerebral ischemia and hypoxia induce HIF-1*α* production, comprehensively regulate the upregulation of VEGF expression, bind VEGF to VEGFR2, and activate Notch signaling pathway through intercellular stimulatory signals. The relationship between Notch signaling pathway molecules and VEGFR interaction is that they work together to promote the formation of new blood vessels. There is no divergent field for the time being. The novelty of this study is that by detecting the changes of HIF-1*α* in the ischemic cerebral cortex, it starts the main process of angiogenesis by regulating the corresponding downstream target genes and has an important effect on angiogenesis after ischemia. By detecting the changes of Hes1+VIII factor expression in the ischemic area, the HIF-1-VEGF-Notch signaling pathway becomes the main regulatory pathway in the process of angiogenesis after ischemia.

In summary, by detecting changes in Hesl+VII factor expression in ischemic areas, the results indicate that ischemia and hypoxia activate the HIF-l, and with the increase in HIF-1 expression, the proliferation of vascular endothelial cells is increased, effectively contributing to neovascularization and making the HIF-1 a major regulatory pathway in the process of postischemic vascular neogenesis.

## Figures and Tables

**Figure 1:** The number of HIF-1*α* positive cells. All HIF-1 expression data in this study were entered by the author into Excel software, and the statistical processing software was calculated by SPSS25.0, expressed as mean ± standard deviation, and found by independent samples *t*-test. In the brain the number of HIF-1*α* positive cells in the cortex increased only slightly after 6 h and 1 d after ischemia-reperfusion, and the number of HIF-1*α* positive cells after 6 h and 1 d was not significantly different from the control group (*P* > 0.05). The number of HIF-1*α* positive cells increased significantly when compared with the control group, and the difference was statistically significant (*P* < 0.05).

**Figure 2:** Expression of VEGFR2. All HIF-1 expression data in this study were entered by the author into Excel software, and the statistical processing software was calculated by SPSS25.0, expressed as mean ± standard deviation, and found by independent samples *t*-test. The number of VEGFR2-positive cells in the cortex increased slightly after 6 h and 1 d of perfusion. There was no significant difference in the number of VEGFR2-positive cells after 6 h and 1d compared with the control group (*P* > 0.05). However, the number of VEGFR2-positive cells increased significantly at 3 d. Compared with the control group, there was a significant difference with statistical significance (*P* < 0.05).

**Figure 3:** Changes in microvessel density. All changes in microvessel density in this study were entered by the author into excel software, and the statistical processing software was calculated by SPSS25.0, expressed as mean ± standard deviation, and found by independent samples *t*-test. The number of Hes1+factor VIII positive cells in the ischemic cortex after 6 hours of perfusion was lower than normal, and there was a statistically significant difference between the control group and the 6 h group by *t*-test (*P* <0.05). The number of factor-positive cells increased significantly, and there was a significant difference compared with the control group, with statistical significance (*P* <0.05).

**Figure 4:** Changes in microvessel density. All changes in this study were entered by the author into Excel software, and the statistical processing software was calculated using SPSS 25.0, expressed as mean ± standard deviation, independent sample *t*-test. The expression of notch1 protein in the cerebral cortex at 6 h, 1 d, and 3 d after ischemia showed a gradual increasing trend, reaching a peak at 3 d, while the expression of Hes1 protein showed a process of first decreasing and then increasing. At 6 h after ischemia, the expression of Hes1 protein was significantly lower than the normal level, and the protein expression level increased significantly at 1 d and 3 d.

## Data Availability

No data were used to support this study.
